The article "Percutaneous Endoscopic Lumbar Discectomy for the Treatment of Recurrent Lumbar Disc Herniation: A Meta-analysis" was published in 2022. Journal: Biomed Res Int.

# Percutaneous Endoscopic Lumbar Discectomy for the Treatment of Recurrent Lumbar Disc Herniation: A Meta-analysis

**DOI:** 10.1155/2022/6488674

**Published:** 2022-09-10

**Authors:** Ke Zhao, Lin-Da Li, Tong-Tong Li, Yong Xiong

**Affiliations:** ^1^College of Acupuncture and Orthopedics, Hubei University of Chinese Medicine, Wuhan, Hubei 430061, China; ^2^Hubei Provincial Hospital of Traditional Chinese Medicine, Wuhan 430061, China

## Abstract

**Objective:**

To evaluate the incidence and safety of clinical complications associated with percutaneous endoscopic lumbar discectomy (PELD) for the treatment of recurrent lumbar disc herniation (RLDH) by meta-analysis.

**Methods:**

PubMed, Embase, The Cochrane Library, and Web of Science electronic databases were searched for clinical studies on complications related to the treatment of RLDH with PELD. The search time extended from the databases' inception until May 2021. RevMan5.4 software was used for meta-analysis after two researchers independently scanned the literature, gathered data, and assessed the bias risk of the included studies.

**Results:**

A total of 8 clinical studies, including 1 randomized controlled trial and 7 cohort studies including 906 individuals, were included. According to the results of the meta-analysis, the overall complications (OR = 0.18, 95% CI: 0.04-0.83, *p* = 0.03) and dural tear rates (OR = 0.11, 95% CI: 0.01-0.92, *p* = 0.04) of PELD were lower than those of traditional fenestration nucleus pulposus removal. Moreover, the PELD group had a greater recurrence rate compared to the MIS-TLIF group (OR = 19.71, 95% CI: 3.68-105.62, *p* = 0.0005), and the difference was statistically significant. However, compared with MED and MIS-TLIF, there were no significant differences in the incidence of overall complications, dural tear, nerve root injury, and incomplete nucleus pulposus removal (*P* > 0.05).

**Conclusion:**

PELD is an effective and safe method for the treatment of recurrent lumbar disc herniation, with a lower incidence of complications and higher safety profile than traditional fenestration nucleus pulposus removal.

## 1. Introduction

Recurrent lumbar disc herniation (RLDH) is a disorder in which the nucleus pulposus of the lumbar disc herniates ipsilateral or contralateral to the original segment after previous surgical treatment for LDH, resulting in back and leg pain [1, 2]. As the number of surgical interventions increases, similarly, the incidence of postoperative recurrence of LDH increases; the incidence of postoperative recurrence varies, with an overall range of 3% to 18% [3]. RLDH is typically defined as a “painless period” of more than 6 months following the first lumbar discectomy, during which the intervertebral disc tissue of the original operative segment protrudes again on the operative side or contralateral side [4]. Surgical intervention is indicated for patients with a definite diagnosis of RLDH if the pain is not relieved after a period of conservative treatment. However, the scar tissue in the surgical area following the first operation increases the difficulty of repeated discectomy and increases the risk of permanent nerve root injury, dural tear with cerebrospinal fluid leakage, and sunburn complications [5]. Meanwhile, further resection of the posterior structure may increase the likelihood of lumbar segmental instability [6]. The ongoing advancements and maturation in percutaneous endoscopic lumbar discectomy (PELD) offer a novel approach for the therapy of RLDH. Compared with other operations, its advantages such as less trauma, faster recovery, less bleeding, and favorable curative effect have been recognized by spinal surgeons. However, some studies have recently reported the occurrence of clinical complications of PELD for the treatment of RLDH; therefore, it is imperative to conduct a thorough meta-analysis to assess the safety of PELD in the treatment of RLDH, so as to further provide an evidence-based foundation for clinical application.

## 2. Materials and Methods

### 2.1. Literature Search Strategy

The PubMed, Embase, The Cochrane Library, and Web of Science databases were electronically searched, and clinical studies related to the complications of PELD for the therapy for RLDH were collected until May 2021. In addition, the references included in the research were manually searched for supplementary and pertinent literature. The keyword researched including “recurrent,” “intervertebral disc displacement,” “disc herniation,” “microdiscectomy,” “percutaneous lumbar discectomy,” “endoscopy discectomy,” “transforaminal lumbar discectomy,” “endoscopic transforaminal diskectomy,” “endoscopic interlaminar discectomy,” and “minimally invasive discectomy.”

### 2.2. Study Inclusion Criteria and Exclusion Criteria

The following are the inclusion criteria: (1) Study design includes randomized controlled trials (RCT), nonrandomized controlled trials, cohort studies, and case-control studies; (2) patients in the study experienced recurrent symptoms more than 6 months following the first lumbar discectomy, with reoccurrence of low back pain with lower limb nerve root pain and numbness. Moreover, lumbar intervertebral disc herniation of the same segment was confirmed by imaging techniques. (3) In the observation group, patients with RLDH were treated with PELD. The surgical methods included percutaneous endoscopic discectomy via the foraminal or interlaminar approach. In the control group, patients received traditional lamina fenestration discectomy, posterior lumbar interbody fusion (PLIF), posterior transforaminal lumbar interbody fusion (TLIF), MIS-TLIF, or posterior microendoscopic discectomy (MED). (4) The primary outcomes included the incidence of total complications, dural tear, intervertebral space infection, nerve root injury, recurrence, and incomplete removal of nucleus pulposus. The following factors determined exclusion: (1) the study included patients with spinal deformity, apparent lumbar instability, lumbar spinal stenosis, spinal infection, tumor or tuberculosis, blood coagulation dysfunction, severe cardiopulmonary dysfunction, and other diseases; (2) non-English literature; (3) duplicated publications from the same hospital or research center; (4) incomplete or missing data, the author of the original study cannot be contacted.

### 2.3. Data Extraction

Two authors extracted pertinent data separately from eligible studies and cross-checked them. In the event of disagreements, they were resolved through dialogue or collaboration with an outside party. The contents of data extraction included (1) first author, publication time, study design, baseline characteristics of subjects, type of operation, and follow-up time. (2) Clinical outcome indices included overall incidence of complications, including postoperative sensory abnormality, dural tear rate, postoperative infection, and so on.

### 2.4. Methodological Quality

The two authors analyzed the risk of bias in the research independently and cross-checked their findings. For case-control and cohort studies, the Newcastle-Ottawa scale (NOS) [7] was used; for randomized controlled trials, the Cochrane manual-recommended RCT bias risk assessment tool [8] was used to evaluate the bias risk.

### 2.5. Statistical Analysis

The meta-analysis was performed using the Review Manager (RevMan version 5.4) software. The mean difference or standard deviation of the mean difference was used as the effect index for continuous variables, while the odds ratio (OR) was utilized for dichotomous variables. The estimated value and 95% CI of each effect quantity were calculated. Chi-square was utilized to examine statistical heterogeneity among the research results and was combined with the *I*^2^ test to quantitatively estimate the magnitude of heterogeneity. If *p* > 0.1 and *I*^2^ < 50%, the fixed effect model was used for the meta-analysis; if *p* ≤ 0.1 or *I*^2^ ≥ 50%, the random effect model was used for meta-analysis after excluding the studies with high heterogeneity. *α* = 0.05 was considered statistically significant.

## 3. Result

### 3.1. Identification of Eligible Studies

A total of 848 studies were obtained through an electronic database search.  Figure 1 illustrates the literature screening procedure. After preliminary examination, rescreening, and finally including 8 articles comprising 1 RCT study and 7 cohort studies [9–16], there were a total of 906 participants in this study.

### 3.2. Characteristics of Included Studies

There was no statistically significant difference between gender, age, and other baseline characteristics of patients included in the literature (Table 1).

### 3.3. Quality of Included Studies

For the 7 included cohort studies, the NOS bias risk score was 6~9 (Table 2). For the included RCT study, the bias risk was assessed according to the Cochrane manual (Table 3).

### 3.4. Meta-analysis Outcomes

#### 3.4.1. Overall Incidence of Complications

A total of 8 studies reported complications. Of the 436 patients in the PELD group, 25 had complications, representing an incidence of 5.73%. The outcomes of the random effect model meta-analysis revealed that the overall incidence of complications in the PELD group was significantly lower than that in the open lumbar surgery group (OR = 0.18, 95% CI: 0.04-0.83, *p* = 0.03). Compared with the MED and MIS-TLIF groups, PELD group incidence was lower than MED group incidence, However, the disparity was not statistically significant (Figure 2).

#### 3.4.2. Dural Tear

There were 6 studies that reported the incidence of intraoperative dural tears. Among the 394 patients in the PELD group, 3 suffered from dural tears (0.76%). The results of the meta-analysis of the fixed effect model exposed that the incidence of dural tears in the PELD group was lower than that in the open lumbar surgery group (OR = 0.11, 95% CI: 0.01-0.92, *p* = 0.04). The incidence of dural tear was quantitatively reduced in the PELD group compared to the MIS-TLIF group, but the meta-analysis revealed no significant difference between the two groups (Figure 3).

#### 3.4.3. Nerve Root Injury

Five studies reported the occurrence of nerve root injury. Of the 362 patients who underwent PELD, 7 experienced complications (1.93%). The meta-analysis with a fixed effect model revealed that the incidence of nerve root injury was lower in the PELD group than in the MED group, but the difference was not statistically significant. Compared with the MIS-TLIF group, the incidence of nerve root injury in the PELD group was higher, but the difference was not statistically significant (Figure 4).

#### 3.4.4. Recurrence Rate

A total of 6 studies investigated the incidence of postoperative recurrence; of the 394 patients who underwent PELD, 37 cases recurred, with an incidence of 9.39%. The meta-analysis using a fixed effect model demonstrated that the recurrence rate in the PELD group was lower than that in the open lumbar surgery group, but the difference was not statistically significant. Likewise, compared with the MED group, the incidence of recurrence in the PELD group was higher. However, no statistical difference existed between the two groups. More importantly, the results revealed that the PELD group had a greater recurrence rate than the MIS-TLIF group, and the difference was statistically significant (OR = 19.71, 95% CI: 3.68-105.62, *p* = 0.0005) (Figure 5).

#### 3.4.5. Incomplete Nucleus Pulposus Extirpation

Only 2 articles reported the incidence of incomplete removal of nucleus pulposus in the PELD and open lumbar surgery groups. Complications occurred in 2 cases (1.9%) in the PELD group and 4 cases (5.7%) in the open lumbar surgery group. The fixed effect model meta-analysis revealed that the PELD group had a lower rate of incomplete nucleus pulposus removal than the open lumbar surgery group, but the difference was not statistically significant (OR = 0.71, 95% CI: 0.14-3.49, *p* = 0.67) (Figure 6).

#### 3.4.6. Postoperative Infection

Two articles documented the incidence of postoperative infection in the PELD and open lumbar surgery groups. There were no cases of postoperative infection in the PELD group. The results of the fixed effect model meta-analysis revealed no statistically significant difference between the PELD and open lumbar surgery groups (Figure 7).

### 3.5. Sensitivity Analysis

The sensitivity of the main index of overall complications was analyzed by excluding individual studies from the meta-analysis, and the results of the meta-analysis were not significantly altered, suggesting a low heterogeneity in the meta-analysis.

### 3.6. Publication Bias

From the funnel chart employed to test the publication bias in the outcome index of overall complications, it can be deduced that the distribution of each study is symmetrical, demonstrating a low likelihood of publication bias (Figure 8).

## 4. Discussion

Laminectomy was long regarded as the treatment of choice for LDH, but several studies have reported that the recurrence rate following LDH ranged from 5% to 18% [17], while the reoperation rate was 13.9% [18]. Repeated fenestration of the nucleus pulposus is regarded as the therapy of choice for recurrent lumbar disc herniation following the initial surgical procedure [19, 20]. However, after RLDH revision surgery, the incidence of complications including nerve root injury, dural tear, and postoperative sensory abnormalities increased, as well as the degeneration of spinal motor units such as facet joints [21]. During the past decade, numerous minimally invasive operations have been developed for the treatment of RLDH, including microscopic disc removal, discoscopic nucleus pulposus extraction (MED), collagenase injection combined with targeted radiofrequency, minimally invasive (Quadrant channel expansion system), and spinal endoscopic techniques, and the clinical outcomes are comparable to that of traditional open surgery [10]. PELD is an established minimally invasive surgical treatment. With advancements in PELD for the treatment of LDH, more and more spinal surgeons have recognized that complications related to scar tissue and posterior structure trauma can be solved by PELD. Yeung and Tsou [22] introduced PELD for the treatment of RLDH first time and accomplished satisfactory results with “intradiscal-extradiscal” clearance of herniated nucleus pulposus tissues from the intervertebral space under direct vision. Since then, increasingly more studies have discovered that the application of PELD for RLDH provides a minimally invasive and effective treatment alternative for RLDH patients [23].

Earlier researches have validated that the clinical efficacy of PELD for the treatment of RLDH is similar to that of other revision surgeries, and some studies have described that its clinical efficacy is actually superior to that of other revision surgeries [24–26]. As per studies, epidural and perineural scar tissue heightens the danger of nerve root injury as well as intraoperative dural rupture [25]. According to previous studies, the incidence of dural tear in lumbar discectomy is 6.9%-20%, which has an adverse impact on the clinical outcomes of the operation [27]. Herein, 11.69% of patients undergoing conventional windowed nucleus pulposectomy suffered from dural tears, compared to no dural tears in patients of the PELD group. In PELD surgery, scar tissue can be selectively excised from nerve tissue under a microscope, and residual scar tissue can be employed as a protective layer of nerve tissue, which may be the reason behind the low incidence of dural injury in patients undergoing PELD.

Reviewing the related literature [28] corroborated that the incidence of nerve root adhesion following transforaminal PELD is low, and patients with uncalcified disc herniation, nonsevere neurological defect, confirmed diagnosis of sciatica, and symptom duration less than 3 months after recurrence should be prioritized. Nevertheless, the interlaminar approach remains the optimal treatment for patients with large intraspinal prolapse, high prolapse, calcified disc herniation, L5/S1 disc herniation with the high iliac spine, and severe lumbar intervertebral foramen osseous stenosis. The transforaminal approach or interlaminar approach for PELD can effectively avoid scar tissue resulting from the first posterior operation, thus limiting the degradation of the spine's posterior structure without compromising its stability and minimizing the incidence of severe complications such as nerve injury and dural tear caused by traditional reoperation to separate the posterior scar tissue.

Prior studies have reported that the recurrence rate of patients who had undergone MED, PELD, or open discectomy and required revision PELD surgery was 4.62%~7.69% [26]. In this study, the recurrence rate of PELD for the treatment of RLDH was 8.37%. The results demonstrated that MIS-TLIF had a much lower recurrence rate than PELD, which is consistent with the findings of prior research [24]. A few studies have also pointed out that the effect of surgery after the recurrence of intervertebral disc herniation relates to the type of the initial operation [29]. Moreover, given the steep learning curve of PELD, many surgeons lack the experience to estimate the number of intervertebral disc materials to be removed during surgery, leaving the possibility of residual nucleus pulposus. However, this study found that the rate of residual nucleus pulposus following PELD (3.33%) was lower than that of traditional windowing surgery (5.19%).

Eight studies were examined for this study, and the bias risk assessment results of the various design types indicated that the studies were of excellent quality. Sensitivity analysis was utilized to exclude studies one by one from the meta-analysis. Lastly, the funnel chart displayed that the possibility of publication bias was small, showing the reliability of the results of this meta-analysis.

The following are the limitations of this meta-analysis: (1) sample sizes in individual research were modest, which impacted the extrapolation of the results; (2) only a single randomized controlled trial was included in the analysis, and the allocation of hidden and blind methods was not mentioned; hence, the likelihood of implementation and measurement bias is higher; (3) the duration of follow-up considerably varied, and the number of cases developing postoperative complications in the PELD and MED groups was relatively low. Therefore, the long-term complication rate and recurrence rate of PELD for the treatment of RLDH require additional study.

To sum up, compared with traditional lamina fenestration, PELD has a lower incidence of complications and a higher safety profile for the treatment of RLDH. Nevertheless, PELD has a similar incidence of complications for the treatment of RLDH compared to MED and MIS-TLIF. Therefore, we postulate that PELD is an efficient and safe surgical technique for treating individuals with RLDH without imaging lumbar instability. As a result of the restricted number of included studies, the aforementioned conclusions require additional validation by high-quality, large sample size studies.

## Figures and Tables

**Figure 1:** Flow chart of the literature search.

**Figure 2:** Forest chart of the overall incidence of complications.

**Figure 3:** Forest chart of the incidence of dural tears.

**Figure 4:** Forest chart of the incidence of nerve root injury.

**Figure 5:** Forest chart of postoperative recurrence rate.

**Figure 6:** Forest chart of the incidence of incomplete nucleus pulposus excision.

**Figure 7:** Forest chart of the incidence of postoperative infection.

**Figure 8:** Funnel plot of the overall complication rate.

**Table 1:** The basic characteristics of the included literature.

Author, year	Design	Operation type		Sample size (male/female)		Mean age (years)		Follow-up (months)	
		Observe group	Control group	Observe group	Control group	Observe group	Control group	Observe group	Control group
Chen (2015)[1]	RCS	PELD	NPLW	18 (12/6)	25 (14/11)	57.40 ± 12.40	54.90 ± 16.60	NR	NR
Lee (2009)[6]	RCS	PELD	NPLW	25 (16/9)	29 (22/7)	42.0 ± 11.4	47.7 ± 12.2	34.0 ± 4.4	34.3 ± 4.6
Lee (2018)[12]	RCS	PELD	NPLW	35 (25/10)	48 (30/18)	52.20 ± 12.87	50.13 ± 11.56	24.17 ± 11.83	23.65 ± 7.94
Liu (2017)[13]	RCS	PELD	MIS-TLIF	209 (110/99)	192 (92/100)	57.2	55.9	43.7	45.3
Ruetten (2009)[9]	RCT	PELD	MED	50	50	39	39	24	24
Wang (2020)[16]	RCS	PELD	MIS-TLIF	24 (14/10)	22 (14/8)	49.25 ± 13.95	56.00 ± 7.76	12	12
Yao (2017)[14]	RCS	PELD	MED/MIS-TLIF	28 (18/10)	20 (11/9)/26 (13/13)	53.68 ± 17.70	51.05 ± 16.38/51.62 ± 10.04	12	12
Yao (2017)[14]	RCS	PELD	MIS-TLIF	47 (72.34%)	58 (72.41%)	47.91 ± 14.77	46.76 ± 12.37	12	12

Note: RCT: randomized controlled trial; PCS: prospective cohort study; RCS: retrospective cohort study; PELD: Percutaneous endoscopic lumbar discectomy; NPLW: nucleus pulpotomy by lamina window; MED: microendoscopic discectomy; MIS-TLIF: minimally invasive transforaminal lumbar interbody fusion; NR: not reported.

**Table 2:** Results of risk assessment of bias in cohort studies.

Study	Selection	Comparability	Outcome	Total
Chen (2015)[10]	★★★★	★	★	6
Lee (2009)[6]	★★★★	★★	★★★	9
Lee (2018)[12]	★★★★	★★	★★★	9
Liu (2017)[13]	★★★★	★★	★★★	9
Wang (2020)[16]	★★★★	★★	★★★	9
Yao (2017)[14]	★★★★	★	★★★	8
Yao (2017)[14]	★★★★	★	★★★	8

**Table 3:** RCT bias risk assessment results.

Included study	Random method	Distribution and hidden	Participant blind method	Blind method of outcome evaluation	Integrity of outcome data	Publish research results selectively	Other sources of bias
Ruetten (2009)[9]	Random number table	Dimness	Single blind	Dimness	No lost of follow-up	No	Dimness

## Data Availability

The data that support the findings of this study are openly available in PubMed, Embase, The Cochrane Library, and Web of Science electronic databases.
